# Murine hypothalamic destruction with vascular cell apoptosis subsequent to combined administration of human papilloma virus vaccine and pertussis toxin

**DOI:** 10.1038/srep36943

**Published:** 2016-11-11

**Authors:** Satoko Aratani, Hidetoshi Fujita, Yoshiyuki Kuroiwa, Chie Usui, Shumpei Yokota, Ikuro Nakamura, Kusuki Nishioka, Toshihiro Nakajima

**Affiliations:** 1 Institute of Medical Science, Tokyo Medical University, Shinjuku-ku, Tokyo, Japan; 2 Department of Future Medical Science, Tokyo Medical University, Shinjuku-ku, Tokyo, Japan; 3 Physician, Student and Researcher Support Center, Tokyo Medical University, Shinjuku-ku, Tokyo, Japan; 4 Department of Neurology and Stroke Center, Mizonokuchi Hospital, Teikyo University School of Medicine, Kawasaki, Japan; 5 Department of Psychiatry, Juntendo University Nerima Hospital, Nerima-ku, Tokyo, Japan; 6 Japan Medical Research Foundation, Chiyoda-ku, Tokyo, Japan; 7 Integrated Gene Editing Section (iGES), Tokyo Medical University Hospital, Shinjuku-ku, Tokyo, Japan

## Abstract

Vaccination is the most powerful way to prevent human beings from contracting infectious diseases including viruses. In the case of the human papillomavirus (HPV) vaccine, an unexpectedly novel disease entity, HPV vaccination associated neuro-immunopathetic syndrome (HANS), has been reported and remains to be carefully verified. To elucidate the mechanism of HANS, we applied a strategy similar to the active experimental autoimmune encephalitis (EAE) model - one of the most popular animal models used to induce maximum immunological change in the central nervous system. Surprisingly, mice vaccinated with pertussis toxin showed neurological phenotypes that include low responsiveness of the tail reflex and locomotive mobility. Pathological analyses revealed the damage to the hypothalamus and circumventricular regions around the third ventricle, and these regions contained apoptotic vascular endothelial cells. These data suggested that HPV-vaccinated donners that are susceptible to the HPV vaccine might develop HANS under certain environmental factors. These results will give us the new insight into the murine pathological model of HANS and help us to find a way to treat of patients suffering from HANS.

There is a long history of the fight between human beings and invasive bacteria and viruses. In the 19^th^ century, Edward Jenner successfully developed and administrated the first vaccine to humans to protect against smallpox. In the 20^th^ century Walther Fleming’s discovery of penicillin, made it possible to directly kill bacteria. These two therapeutic developments have not only given us a way to prevent and treat infectious diseases, but have also led to a tremendous improvement in human welfare.

Cervical cancer is the most common type of cancer in women and is the cancer associated with the most death in women aged younger than 44. Because infection with human papilloma viruses (HPVs) is necessary for the occurrence of cervical cancer, protection from HPV is effective in avoiding the disease^1^,^2^. There are 40 types of HPVs which can infect anogenital epithelium in humans, and 15 types of the virus are associated with cervical cancer^3^,^4^. In general, vaccine is designated to prevent against infectious diseases. To prevent HPV infection, two prophylactic vaccines have been developed; a quadrivalent vaccine (Gardasil^®^; Merck & Co., USA) against L1-like virus particles to HPV types 6, 11, 16 and 18^5^, and a bivalent HPV vaccine (Cervarix^®^; Glaxo Smith Kline, London) against types 16 and 18, which are thought to be the most frequent of the 15 types associated with cervical cancer. Clinical trials revealed both Gardasil and Cervarix to be safe and effective against cervical cancer^6^; thus, the two vaccines were introduced for administration in 2006 with approximately 175 million doses being distributed worldwide since then.

Like Janus’ mirror, however, immunization and vaccination have two different aspects and some kinds of strongly evoked immune reactions are thought to result in significant adverse reactions. For example, a few cases have determined vaccine to be the cause of abnormal and dysregulated host-reactions, resulting in such as systemic fever, local pain at the injection site, Guillain-Barré syndrome-like neurological deficit, and autoimmune-like symptoms and so on. To evoke a full- and adequate immunological reaction, vaccines include aluminum adjuvant in addition to virus-like particles as antigens. Chronic stimulation of the immune system by adjuvants can result in an autoimmune disease characterized by myalgia, arthralgia, chronic fatigue, and neurological manifestations - appropriately named the autoimmune/inflammatory syndrome induced by adjuvants (ASIA)^7^,^8^. According to the HPV vaccination, there are two recent well-documented review articles. Palmieri B. *et al* reported the occurrence of severe somatoform and dysautonomic syndromes after HPV vaccination^9^ and Brinth L. *et al*. also described the onset of autonomic dysfunction after the quadrivalent vaccination^10^. Both reviews clearly indicated the presence of unique adverse reactions associated with the HPV vaccination including headache, fatigue, depression, cognitive dysfunctions, uncontrollable and involuntary movement, and limb weakness. For these clinical manifestations, we have coined these reactions as human papillomavirus vaccination-associated neuro-immunopathic syndrome (HANS) and proposed diagnostic criteria. HANS syndrome is thought to consist of four clinical domains; (i) autonomic, endocrine and inflammatory symptoms; (ii) cognitive and emotional symptoms; (iii) environmental hypersensitivity and pain symptoms and (iv) locomotion and motor symptoms^11^,^12^. Several clinical studies on HANS symptoms have also shown that the HPV vaccines may influence the central nervous system (CNS)^10^,^13^,^14^,^15^.

In this study, to better understand the molecular mechanisms of HANS, we first attempt to establish an animal model of the syndrome. We then analyzed the pathological lesions of the murine HANS model by focusing on the CNS.

## Results

### HPV vaccine Administration

To assess the neurophysiological effects of the HPV vaccine, forty eight female mice were either immunized with Gardasil or given phosphate-buffered saline (PBS) as a control (Fig. 1-a). Pertussis toxin (Ptx) was administrated subsequent to the vaccination to facilitate the access of the vaccine to the CNS via modulation of the blood-brain barrier (BBB)^16^. As a control for autoimmune encephalomyelitis, myelin oligodendrocyte glycoprotein (MOG)_35-55_ was used^17^. Administration of PBS or Ptx had no effect (group 1, 2), and disruption of BBB by Ptx itself was confirmed to have no effect. Mice in group 5 and 6 belonged to the experimental autoimmune encephalitis (EAE) groups. Mice in the group 6 that had received MOG and Ptx showed paralyzed tails within 2 weeks, and various neurological symptoms, such as hind limb paresis after 3 weeks. Mice in the group 5, had received MOG without toxin administration, also revealed neurological symptoms, which was advanced more slowly than group 6 as reported previously^18^. Mice in group 3 and 4 belonged to the Gardasil treatment groups. After a third injection of the vaccine (4 weeks from first immunization), three out of 16 mice in group 4, which were treated with Gardasil and Ptx, presented the tail with reduced tension and significantly weakness movement (Fig. 1-b). Motor disability was graded by use of an EAE score (scale, 0–6)^19^. Although the symptomatic severity varied, over 50% of mice (12/21) showed similar motor dysfunctions, including tail drop as shown in Fig. 1-a, over the course of the study. Two of the 14 mice with sequential immunization with Gardasil alone administration (group 3) exhibited milder motor dysfunctions compared with the combined treatment group with Gardasil and Ptx (Fig. 1-b,c). We confirmed the behavior of these mice by horizontal bar test and Kondziela’s inverted screen test^20^,^21^. Significant decrease of motor coordination was observed in the combined treatment group with Gardasil and Ptx, compared to control group. By contrast, there were no differences in the muscular strength between these groups, (Supplemental Figure 1). Altogether, these results suggest that combined administration of HPV vaccine and Ptx could induce the damage to the murine CNS.

### Pathological analyses

For further investigation of the neuropathological lesions associated with HPV vaccination, histological analyses of the brain were performed. Overall, the groups exhibited no differences in brain size or weight. Serial brain dissections were obtained 12 weeks after the first immunization, and they underwent hematoxylin and eosin (H&E) staining and Klüver-Barrera (KB) staining. H&E staining revealed contracted third ventricles in mice treated with Gardasil and Ptx (Fig. 2-a upper). On the other hand, mice that had undergone EAE, showing paralysis of the tail and hind limbs, did not appear to have narrowed third ventricles. Similarly, treatment with Ptx or Gardasil alone did not lead to third ventricular stenosis. Morphological differences were also not detected in the cerebellum, spinal cord, cortex among vehicle of mice treated with Gardasil alone, Ptx and Gardasil with Ptx (Group 1, 2, 3 and 4). Serial sections of the forebrains from mice treated with Gardasil and Ptx were stained and revealed that the third ventricle was remarkably narrowed over a wide range of the forebrain from anterior to posterior portion (Fig. 2-b). Together, our analyses suggest that treatment with HPV vaccine could affect the ventricular size and cerebrospinal fluid (CSF) pressure.

To confirm the relationship between effects of HPV vaccine on motor function and histological changes, differences around the third ventricle were compared among mice treated with Gardasil and Ptx. In the vaccine-treated group, the third ventricle was narrowed in all mice showing tail drops. Additionally, the extent of third ventricle narrowing seemed to be corresponding with the severity of disruptions to tail tonus (Fig. 2-d). In H&E staining of the paraventricular hypothalamic nuclei (PVN), the dorsomedial hypothalamic nuclei (DMH) and the arcuate nuclei from mice treated with Gardasil and Ptx, indicated less stained nuclei than mice in other groups (Fig. 2-b,d). KB staining of the same structure also revealed a decrease in the number of nuclei and Nissl bodies (Fig. 2-c,d). In addition, we confirmed effects on the inflammation by HPV vaccine and Ptx. The filtration of lymphocytes into forebrain was not observed (Fig. 2-b).

### Induction of Apoptosis in the Circumventricular Regions

The decrease in the number of cells led us to assess the association between HPV vaccination and apoptosis in the forebrain. In order to do this, we performed the TUNEL assay on sections of the forebrain. In sections obtained from vehicle- and Ptx-treated animals, we found a limited number of TUNEL-positive cells with labelled nuclei - confirming that Ptx alone did not induce apoptosis. Meanwhile, greater numbers of TUNEL-positive cells were found in the thalamus and the hypothalamus obtained mice treated with Gardasil and Ptx (Fig. 3). In fact, seven times more TUNEL-positive cells were observed in mice treated Gardasil and Ptx, while four times more apoptotic cells were found in mice treated with Gardasil alone than that apoptotic cells in vehicle mice. In particular, the number of labelled cells was greater around the third ventricle and at the vessels in PVN and DMH. Together, these data support an association between apoptosis and the damage to murine neural structures caused administration of HPV vaccine and Ptx.

### Identification of Apoptotic Cells

Next, we sought to determine which types of cells were affected by apoptosis. Since apoptotic cells were observed around vessels, we labeled sections using markers for vascular endothelial cells, pericytes and astrocytes. CD31-expressing cells were consistent with apoptotic cells bound to vessels (Fig. 4), while cells expressing NG2- or GFAP were not stained. There results indicate that the HPV vaccine induced vascular endothelial cell apoptosis.

### Neurotransmission in circumventricular regions

Finally, for further the understanding of neuronal damage in combined administration of HPV vaccine and Ptx mice, we assessed the interneuron subtypes in circumventricular regions (Fig. 5). As a result of immuno-staining, tyrosine hydroxylase (TH) was increased in PVN, particularly arcuate nuclei, of mice treated with Gardasil and Ptx compared with the area of vehicle mice. On the other hand, glutamic acid decarboxylase (GAD) 67 and gamma-aminobutyric acid (GABA) was decreased in PVN. The expression of glutamine synthetase, choline acetyltransferase was not changed. These results indicated that dopaminergic neurons were increased in the arcuate nuclei, while GABAergic neurons were reduced.

## Discussion

In this study, we demonstrated that the combined administration of Gardasil and Ptx induced of poor tail movement and low locomotive mobility. In addition, vaccination did not have effect on the muscular strength. Neuropathological observation reveals the following results; (1) structural damage to PVN, DMH, (2) the third ventricular atresia, (3) an increase in apoptosis around cavities of the thalamus and the hypothalamus; vascular endothelial cells in the hypothalamus were especially affected, and (4) increasing TH synthesis and decreasing GABA synthesis in the arcuate nuclei.

The low locomotive mobility of mice in group 4 (Fig. 1) was appeared to be derived from disruption of hypothalamic motor networks, since pathological changes were discretely localized at the circumventricular structures (Fig. 2) and their muscle strength was normal. Several animal experiments have highlighted the importance of the hypothalamus for motor command, and indicate that hypothalamic command signals are primarily responsible for the driving of locomotion and that locomotor stepping is mediated by the perifornical and lateral hypothalamus^22^,^23^,^24^, while flight-directed locomotion and escaped jumps are mediated by medial hypothalamus^25^. The hypothalamus has also an important role in integration of neuronal circuitry for motor regulation, with connections to cingulate motor cortex in the limbic system, which project to the spinal cord and red nucleus, and have premotor functions^26^. Since low mobility of the body on locomotive movements can be also seen frequently in patients suffering from HANS, we hypothesize that locomotive impairments in both murine motor phenotype and human HANS are linked to disrupted hypothalamic motor areas.

The cerebral ventricles are filled with CSF and constitute a communicating network connecting cavities^27^. Our data suggest that HPV vaccination may induce vascular endothelial cell apoptosis and may disrupt BBB-CSF barriers. Moreover, the narrowing of the ventricle could have been due to collapse of the barriers between the brain and ventricles, causing CSF to leak out of the brain^28^. CSF is important for maintaining brain homeostasis, and narrowing of the ventricles is often seen in the patients suffering from intracranial hypotension syndrome (ICH). Like the proposed mechanism for the ventricle narrowing observed in the current study, ICH is caused by CSF leakage and low CSF pressure^29^. Interestingly, some of these clinical symptoms are experienced by individuals suffering from HANS, such as orthostatic headache, dizziness, stiffness and so on^30^. Although there is currently no pathological information with regard to of HANS, it could be important to investigate effects of the vaccination on the CSF function and pathological features around the third ventricle in future.

Surprisingly, NK2 Homeobox 1 (Nkx2.1), also known as thyroid-specific transcription factor 1 (TTF-1) -deficient mice have been established and display similar morphological features including structural damage to PVN and DMH and the third ventricular atresia to the vaccine-treated mice in this study. Nkx2.1 has been identified as a transcription factor for thyroid specific factors^31^,^32^, and has also been established as an important factor for early brain development^33^. Nkx2.1 is expressed in the ventral region of the forebrain^34^,^35^. In Nkx2.1-deficient mice, abnormalities are seen in the ventral and medial regions of the hypothalamus, the third ventricle is narrowed, and does not reach to the floor of the diencephalon^36^. Nkx2.1 is also known to be expressed in the hypothalamic region and periventricular areas from early phase of development to adult^35^. Further, Nkx2.1 is thought to play roles in puberty and reproductive function and schizophrenia^35^,^37^,^38^. In humans, Nkx2.1 gene mutations can cause benign hereditary chorea (BHC)^39^,^40^, a disease affecting the brain, lungs and thyroid. Patients with this mutation suffer from chorea, a variety of neurological characteristic, tremor, axial dystonia, and gait disturbance^41^. Taking the literature into account, our current data suggest that the HPV vaccine may disrupt signaling pathway mediated by Nkx2.1 that are expressed in the hypothalamic region. We studied on the neurotransmitters production in order to corroborate pathophysiological correlation of Nkx2.1, since some studies indicated the abnormalities of several neurotransmitters production in Nkx 2.1 deficient-mice in early development^42^, and also in adult mice^35^,^38^. We found similar phenotype of neurotransmitters production in group 4 mice including increase of dopaminergic neurons and reduced GABAergic neurons (Fig. 5). These results may explain the symptom of endocrine system in HANS syndrome.

We have recently revealed the functions of hypothalamus are implicated in HANS by the clinical studies. The endocrine function tests showed the results suggesting hypothalamic dysfunction. HANS disorders are not of psychogenic origin but are derived from neuro-endocrinological disorders of the hypothalamus and its limbic networks^15^. Moreover, evidence has been accumulated which indicates the hypothalamus is concerned in certain elements of behavior/emotion^22^,^24^,^25^ and important for pain regulation^43^,^44^. PVN and DMH, impaired in our murine HANS model, integrally controls autonomic, endocrine, and plays an important role in homeostatic maintenance for those functions. Recent advance in neuroscience has highlighted the importance of the PVN for stress-related synaptic plasticity in the hypothalamus^45^. The DMH and the suprachiasmatic nucleus (SCN) have their roles in circadian control of sleep, and in the brain’s circadian pacemaker, respectively. Excitotoxic DMH lesions reduce circadian rhythms of wakefulness, feeding, and locomotor activity. Therefore, we hypothesize that the likely focus in HANS should be on the hypothalamus and the circumventricular organs around the third ventricle, characterized by leaky blood brain barrier, incidentally those clinical reports about functions of the hypothalamus are consistent with our data using mouse model.

In conclusion, our study revealed that exposure of the CNS to the HPV vaccine can induce neuronal degeneration and result in motor dysfunction in C57/BL6 mice, which were similar to the clinical symptoms associated with the HPV vaccination^9^,^10^. Moreover, co-injection of Ptx induced hypothalamic damages associated with motor dysfunctions at a higher frequency. Namely, it is likely to note the HPV vaccine alone result in weaker phenotype; rather, a mouse strain that is hyper-susceptive strain in its immune reaction (e.g., C57BL6) and the addition of Ptx damaging the BBB are required. There might be hypersensitive girls to HPV vaccine because of unclear predisposing factors and/or environmental concomitant events causing a damage to the BBB probably (similar to the damage that is induced by Ptx in the current study). A variable combination of these factors might result in individual suffering from HANS. Further analyses are required for verifying this possibility; however our data provide the first pathological model of HANS and will allow us in the future to explore a way to treat patients suffering from HANS.

## Methods

### Mice

Nine-week old female C57BL/6 mice were purchased from Sankyo Laboratory (Japan) and used for the vaccination studies. Mice were kept under standard conditions in the animal facility at Tokyo Medical University and were provided with food and water ad libitum. All animal experiments were approved by the Institutional Animal Care and Use Committee of Tokyo Medical University (the approval numbers: s-27050 and s-28039) and performed in accordance with institutional, science community, and national guidelines for animal experimentation.

### Reagents and Antibodies

The antigen for experimental autoimmune encephalomyelitis (EAE) and pertussis toxin (Ptx) were purchased from Hook Laboratories, and the HPV vaccine, Gardasil, was purchased from MSD K.K. The following antibodies were used in this study: anti- NG2, anti-GAD67 and anti-tyrosine hydroxylase antibodies from Merck Millipore (Germany); anti-GFAP, CD31, anti-choline acetyltransferase and anti-Glutamine synthetase from Abcam (Cambridge, UK); anti-GABA antibody from Sigma-Aldrich.

### Vaccination

Groups of 11 week-old female C57BL/6 mice were intramuscularly administrated 100 μl of Gardasil or phosphate-buffered saline (PBS) for a total of five times. Ptx was intraperitoneally administrated 2 and 24 hours after immunization. The Gardasil vaccine or Ptx were administrated at 2- weeks or 4-week intervals, respectively. As a control, EAE was induced with myelin oligodendrocyte glycoprotein 35-55 (MOG_35-55_) followed the manufacturer’s instructions (Hooke Laboratories, USA). Disease severity was evaluated according to the following scores^19^; 0, no abnormality; 1, partially limp tail; 2, loss of tail tonicity; 3, partial hind limb paralysis; 4, complete hind limb paralysis; 5, forelimb paralysis or moribund; 6, death. The most severe symptom of each mouse over the course of the study was evaluated.

### Histology

Mice were anesthetized and transcardially perfused with PBS and 10% formaldehyde in PBS. Brains were then removed, fixed in 10% formaldehyde and embedded in paraffin. Five-micrometer sections were obtained and deparaffinized. For general morphological analyses, hematoxylin and eosin (H&E) and Klüver-Barrera (KB) staining were used. For immunohistochemistry, we performed antigen retrieval by heating sections in citrate buffer and quenched endogenous peroxidase activity by incubating sections in 3% hydrogen peroxide. The sections were blocked with 10% bovine serum albumin (BSA) in PBS and incubated with primary antibodies. After incubation with secondary antibodies conjugated with horseradish peroxidase (HRP), bound antibodies were detected with 3, 3-diaminobenzidine. Stained sections were counterstained with hematoxylin, and all images were obtained using a Nanozoomer (Hamamatsu Photonics, Japan).

### TUNEL Assay

Mouse brains were fixed in 10% formaldehyde in PBS and paraffin embedded. Sections were cut at 5 μM and deparaffinized using a standard procedure. The TUNEL assay was performed using an *in situ* Apoptosis Detection kit (Takara bio Inc. Japan), stained sections were counterstained with hematoxylin.

## Additional Information

**How to cite this article**: Aratani, S. *et al*. Murine hypothalamic destruction with vascular cell apoptosis subsequent to combined administration of human papilloma virus vaccine and pertussis toxin. *Sci. Rep.* **6**, 36943; doi: 10.1038/srep36943 (2016).

**Publisher’s note:** Springer Nature remains neutral with regard to jurisdictional claims in published maps and institutional affiliations.

## Supplementary Material

Supplementary Information

## Figures and Tables

**Figure 1:** Administration of the HPV vaccine to mice. (**a**) Combination of reagents for injection and assessments of mice with neurological symptoms, (**b**) Neurological phenotype associated with vaccination and (**c**) Score of disease severity.

**Figure 2:** Histology of an HPV vaccine-treated brain. (**a**) H&E (upper) and KB (lower) staining of forebrain sections from each group (**b**) H&E staining of serial coronal sections of the forebrain from mice treated with vehicle (upper) and with vaccine and Ptx (lower) (**c**) KB staining of serial coronal sections. Scale bar, 2.5 μm (**d**) H&E (upper) and KB (lower) staining of periventricular sections of the brain from mice with neurological deficits. Scale bar, 500 μm.

**Figure 3:** Detection of apoptosis by TUNEL in mouse brains. Apoptotic cells are indicated by arrows. Scale bar, 500 μm and 50 μm.

**Figure 4:** Immunohistochemistry of the forebrains of vaccinated mice. Forebrain sections from mice treated with vaccine and Ptx were stained with anti-CD31, NG2, and GFAP. Scale bar, 20 μm.

**Figure 5:** Immunostaining of interneuron in circumventricular regions. Sections of forebrain from mice treated with HPV vaccine and Ptx were stained with anti-TH, GAD67, choline acetyltransferase (CA) and glutamine synthetase (GS). Scale bar, 500 μm.
